# Transcription Activation of Rab8A by PEA3 Augments Progression of Esophagus Cancer by Activating the Wnt/*β*-Catenin Signaling Pathway

**DOI:** 10.1155/2023/8143581

**Published:** 2023-02-13

**Authors:** Shusheng Cai, Xiumei Liu, Weiran Gao, Lianhua Ye, Qiming Zhong, Xin Zhang

**Affiliations:** ^1^Department of Digestive System, The First Affiliated Hospital of Jinzhou Medical University, 2 Section 5, Renmin Street, Guta District, 121001 Jinzhou City, Liaoning Province, China; ^2^College of Life Science, Yantai University, 30 Qingquan Road, 264005 Yantai City, Shandong Province, China; ^3^Department of Oncology, The First Affiliated Hospital of Jinzhou Medical University, 2 Section 5, Renmin Street, Guta District, 121001 Jinzhou City, Liaoning Province, China

## Abstract

**Background:**

Rab8A has been reported as an oncogenic gene in breast and cervical cancer. However, the function and molecular mechanism of Rab8A in esophagus cancer has not been reported.

**Methods:**

Rab8A expression was detected by qPCR and western blotting assays, small interference RNA (siRNA) was applied to reduce Rab8A expression, and the biological behaviors of esophagus cancer cells were estimated by cell counting kit-8, colony formation, and transwell and western blotting assays. The transcriptional factor of Rab8A was verified by dual-luciferase assay and chromatin immunoprecipitation assay. The protein expression of key genes in the Wnt/*β*-catenin signaling pathway was determined by western blotting assay. M435-1279 was used to suppress the Wnt/*β*-catenin signaling pathway.

**Results:**

A significant increase of Rab8A expression has been found in esophagus cancer cells. Knockdown of Rab8A suppressed the viability, colony formation, migration, and invasion abilities of esophagus cancer cells and induced apoptosis. PEA3 transcriptionally regulated Rab8A expression and promoted the viability, colony formation, migration, and invasion abilities of esophagus cancer cells and blocked apoptosis, which were diminished by si-Rab8A transfection. Additionally, the expression levels of key genes related to the Wnt/*β*-catenin signaling pathway were strengthened by PEA3 overexpression, which were reduced by si-Rab8A transfection. M435-1279 treatment significantly reduced the viability and colony formation of esophagus cancer cells.

**Conclusions:**

The data showed that Rab8A was transcriptionally regulated by PEA3 and promoted the malignant behaviors of esophagus cancer cells by activating the Wnt/*β*-catenin pathway. The above results indicated that Rab8A may be considered as a promising biomarker for diagnosis and precision treatment in esophagus cancer.

## 1. Introduction

Esophagus cancer is still an integral cause of cancer-related death and has presented a drastic increase of greater than 6-fold in incidence rates worldwide [1]. In China, esophagus cancer is one of the highest morbidity and mortality cancers; nearly 258,000 new cases and 193,000 deaths of esophagus cancer were reported in 2017 [2]. The incidence rate of esophageal cancer varies considerably with location. Despite the great process in the diagnosis and treatment of esophagus cancer, effective biomarkers that contribute to precision diagnosis and therapy are still lacking [3]. Therefore, it is very important to seek for promising biomarker and therapeutic target for the patients with esophagus cancer.

Rab proteins belong to GTPases of the Ras superfamily, and functional damage of Rab8 proteins has been reported to be involved in tumorigenesis, such as Rab1, Rab2A, and Rab8 [4]. Rab8, as a small Ras-related GTPase, was implicated in protein trafficking and secretion [5]. Rab8A and Rab8B were two isoforms of Rab8 in humans, which has 80% homology. Rab8A has been reported to be involved in various cellular functions such as neuronal differentiation and membrane trafficking [6]. Additionally, the effect of Rab8A in cancer has been reported. For example, Rab8A has been found to promote breast cancer progression by elevating surface expression of tropomyosin-related kinase B [7]; Rab8A was reported to promote the growth and metastasis of cervical cancer [8]. However, the function and molecular mechanism of Rab8A in esophagus cancer has not been revealed.

The concept of transcriptional control was put forward half a century ago in bacterial systems [9]. Over the past decade, our knowledge of mammalian regulatory elements and the transcriptional and chromatin regulatory elements that function at these sites has grown considerably [10]. Many different cancers can be caused by mutations in regulatory sequences and transcription factors that interact with these regions [10]. We described the transcriptional regulation of Rab8A in esophagus cancer.

This study was performed to detect the function of Rab8A in esophagus cancer. We estimated the effect of Rab8A depletion on cell proliferation, apoptosis, invasion, and migration. It is of great significance to estimate the molecular pathology to clarify the pathogenesis and disease progression of esophagus cancer patients.

## 2. Materials and Methods

### 2.1. Tissue Collection

A total of 7-paired esophagus cancer specimens and adjacent normal control tissues were collected from esophagus cancer patients undergoing surgery at the First Affiliated Hospital of Jinzhou Medical University. All procedures followed were in accordance with the ethical standards of the responsible committee on human experimentation and with the Helsinki Declaration of 1964 and later versions. Informed consent or substitute for it was obtained from all patients for being included in the study.

### 2.2. Cell Culture and Treatment

Cells (Het-1A, ECA109, TE-1, and KYSE150) were cultured in DMEM medium containing 10% fetal bovine serum (FBS) and placed in a humidified incubator at 37°C in 5% CO_2_. siRab8A-1 (CGGAACTGGATTCGCAACATT) and siRab8A-2 (CGACTATGGAATCAAGTTCAT) were synthesized by Sangon (Shanghai, China) and transfected into TE-1 and KYSE150 cells to reduce Rab8A expression. si-PEA3 (GCTCCGATACTATTATGAGAA) and pcDNA3.1-PEA3 were purchased from Sangon and used for reducing or increasing PEA3 expression. M435-1279 was applied to inhibit the Wnt/*β*-catenin signaling pathway.

### 2.3. RNA Preparation and Real-Time PCR Assay

The whole RNA was extracted by using TRIzol kit (Invitrogen, USA) and reversely transcribed into cDNA by using the cDNA synthesis kit (Beyotime, China). SYBR Green qPCR mix (Beyotime, China) was applied to measure the relative expression of Rab8A in the ABI 7900 system. The expression of Rab8A was calculated by using the 2^-*ΔΔ*Ct^ method. Three independent experiments were carried out to determine Rab8A expression. GAPDH was regarded as the internal reference. The sequences of primers were listed as follows: Rab8A, forward: 5′-CTACGACATCACCAACGAGAAG-3′, Rab8A, reverse: 5′-CATCACACTTGTTCCCGAGTAT-3′; GAPDH, forward: 5′-GCACCGTCAAGGCTGAGAAC-3′, GAPDH, reverse: 5′-TGGTGAAGACGCCAGTGGA-3′.

### 2.4. Western Blotting

RIPA buffer was applied to extract the total protein from cell lysates, and protein concentrations were quantified by a BCA method. Next, the proteins were isolated by 12% SDS-PAGE gel, and then, the proteins were transferred from gels to a PVDF membrane. With sealing in 5% nonfat milk at 25°C for 1 h, the PVDF membrane was followed with the primary antibodies (Rab8A (Abcam, ab188574, 1 : 5000), Bcl-2 (Abcam, ab182858, 1 : 2000), BAK (Abcam, ab243151, 1 : 1000), caspase-3 (Abcam, ab32042, 1 : 500), PEA3 (Abcam, ab236503, 1 : 2000), c-MYC (Abcam, ab19312, 1 : 2000), *β*-catenin (Abcam, ab223075, 1 : 1000), CyclinD1 (Abcam, ab226977, 1 : 1000), Tubulin (Abcam, ab7291, 1 : 5000), and GAPDH (Abcam, ab8245, 1 : 5000)) incubation. Subsequently, the PVDF membrane was blotted with the corresponding secondary antibody for 2 h. Last, the bands were visualized by an enhanced chemiluminescence detection kit. The relative protein expression was normalized to GAPDH or Tubulin.

### 2.5. Cell Viability Detection

KYSE150 and TE-1 cells (2 × 10^3^ cells/well) were implanted into 96-well plates and cultivated to about 80% confluence. After transfection with siRab8A, pcDNA3.1-PEA3, or pcDNA3.1-PEA3+siRab8A, cell counting kit-8 (CCK-8) reagent (10 *μ*L) was put into per well and each well was cultured at 37°C incubator for 90 min. The optical density (OD) value of KYSE150 and TE-1 cells in per well was measured at 450 nm wavelength by a microplate reader.

### 2.6. Cell Cloning Ability Detection

KYSE150 and TE-1 cells were harvested, resuspended in DMEM including 10% FBS, and then implanted in 6-well plates (500 cells each well). After cultivation under standard condition for 2 weeks, the colonies were fixed and stained. Finally, cell colonies were counted and applied for comparisons of colony formation ability.

### 2.7. Transwell Assay

Cell suspension (100 *μ*L) including 2 × 10^4^ cells was added to the upper chamber of a 24-well transwell plate with 8 *μ*m pore polycarbonate filters (Costar, Corning, NY, USA). In the lower chamber, 500 *μ*L of DMEM including 10% FBS was added. After incubation for 24 h, the medium was removed from the upper chamber and cells in each group were erased by a cotton swab. The cells that had migrated to the lower chamber were fixed and stained. Migrating cells were captured under a microscope in five random fields of view. The steps of invasion assay were consistent with the migration assay, except that the upper chamber was precoated with Matrigel. Three independent experiments were performed.

### 2.8. Chromatin Immunoprecipitation (ChIP) Assay

To detect whether PEA3 could bind to the promoter of Rab8A, a ChIP assay was conducted according to the ChIP assay kit procedures (ab500, Abcam). Briefly, the treated cells were collected and lysed. Antibody against Rab8A and IgG was applied for immunoprecipitation. PCR amplification of the precipitated DNA was performed.

### 2.9. Dual-Luciferase Reporter Assay

The potential transcription factor binding sites between Rab8A and PEA3 were generated by online software UCSC (https://genome.ucsc.edu/) and PROMO (http://alggen.lsi.upc.es/). To determine the activity of the Rab8A promoter in the presence of PEA3 overexpression, luciferase assay was performed. First, based on the predicted transcription factor binding sites, wild-type Rab8A (WT-Rab8A), mutant-1 Rab8A (Mut1-Rab8A), and Mut1-Rab8A were amplified and transfected into PGL3 vector. Subsequently, cells were cotransfected with PGL3-Rab8A promoter and PEA3 overexpression vector or the corresponding control vector using Lipofectamine 2000. A total of 48 h following transfection, the relative luciferase activity was measured as normalized to *Renilla* luciferase activity using the Dual-Luciferase® Reporter Assay System (Promega Corporation).

### 2.10. Statistical Analysis

At least three independent experiments were carried out in each group. All experimental data were presented as mean ± standard deviation. The differences were processed by Student's *t*-test (two groups) or one-way analysis of variance (ANOVA) followed by Bonferroni's post hoc test (three or more groups). *P* value less than 0.05 was deemed as a statistically significant difference.

## 3. Results

### 3.1. Rab8A Expression Was Highly Expressed in Esophagus Cancer Samples and Was Significantly Reduced after si-Rab8A Transfection

First, an obvious increase of Rab8A was observed in esophagus cancer cells, including KYSE150, TE-1, and Eca109 cells (Figures 1(a)–1(c)). To further detect the function of Rab8A in esophagus cancer, siRab8A-1 or siRab8A-2 was applied to reduce Rab8A expression in KYSE150 and TE-1 cells. As displayed in Figures 1(d) and 1(e), siRab8A-1 or siRab8A-2 treatment significantly decreased the protein levels of Rab8A in KYSE150 and TE-1 cells.

### 3.2. si-Rab8A Transfection Reduced the Viability, Migration, and Invasion and Induced the Apoptosis of Esophagus Cancer Cells

Next, the OD values, growth ability, apoptosis, migration, and invasion in KYSE150 and TE-1 cells were detected by CCK-8, colony formation, western blotting, and transwell assays, respectively. Results from the CCK-8 assay showed that the OD values in KYSE150 and TE-1 cells were obviously reduced after siRab8A-1 or siRab8A-2 transfection (Figures 2(a) and 2(b)). Moreover, the number of cell clones in KYSE150 and TE-1 cells was obviously decreased after siRab8A-1 or siRab8A-2 transfection (Figures 2(c) and 2(d)). Besides, siRab8A-1 or siRab8A-2 transfection reduced the protein level of Bcl-2 and increased the protein levels of BAK and active caspase-3 (Figures 2(e)–2(h)). Additionally, the number of cell migration and invasion in KYSE150 and TE-1 cells was diminished after siRab8A-1 or siRab8A-2 transfection (Figures 2(i)–2(l)). Therefore, the data suggested that knockdown of Rab8A limited the growth ability, induced apoptosis, and blocked the invasion and migration abilities of KYSE150 and TE-1 cells.

### 3.3. PEA3 Transcriptionally Regulated Rab8A and Affected the Function of Rab8A on Esophagus Cancer Cells

To further explore the molecular mechanism of Rab8A in esophagus cancer cells, the transcriptional factor of Rab8A was captured. PEA3 was discovered to have two binding sites in the promoter region of Rab8A by searching UCSC and PROMO website. Then, luciferase reporter vectors including WT or mutated PEA3 binding sequences (Mut1 and Mut2) were established and cotransfected with corresponding control or PEA3 overexpression (OE) vector into cells. The data showed that PEA3-OE treatment increased luciferase activity in the WT group whereas the luciferase activity in the Mut1 or Mut2 group has no obvious change (Figure 3(a)). Data from ChIP assay showed that depletion of PEA3 reduced Rab8A enrichment compared with that in the si-NC group (Figures 3(b) and 3(c)). Additionally, we also discovered that depletion of PEA3 decreased Rab8A expression in KYSE150 and TE-1 cells, and Rab8A expression was significantly increased after PEA3-OE treatment (Figures 3(d)–3(g)). Moreover, we also detected the protein expression of Rab8A and PEA3 in esophageal cancer tissues. The results showed that Rab8A and PEA3 were both highly expressed in esophageal cancer samples (Figures 3(h) and 3(i)). The above findings revealed that PEA3 could bind to the promoter of Rab8A and regulate Rab8A expression.

### 3.4. The Combined Function of PEA3 and Rab8A in Esophageal Cancer Cells Was Searched

To further investigate the interaction between Rab8A and PEA3, con, PEA3-OE, or PEA3-OE+si-Rab8A was, respectively, transfected into KYSE150 and TE-1 cells. Data from CCK-8 and colony formation assays showed that upregulation of PEA3 elevated the growth ability of KYSE150 and TE-1 cells (Figures 4(a)–4(d)). However, the promoting effect was blocked by si-Rab8A treatment to some extent (Figures 4(a)–4(d)). Moreover, overexpression of PEA3 suppressed the apoptotic ability of KYSE150 and TE-1 cells, whereas the addition of si-Rab8A diminished the phenomena (Figures 4(e)–4(h)). Furthermore, depletion of Rab8A reversed the promoting effect of PEA3-OE on cell migration and invasion (Figures 4(i)–4(l)). These findings suggested that si-Rab8A could antagonize the effect of PEA3-OE on esophageal cancer cell growth, apoptosis, migration, and invasion.

### 3.5. Effect of PEA3/Rab8A on Esophagus Cancer Cells Was Based on the Wnt/*β*-Catenin Signaling Pathway

A growing number of evidence revealed that the Wnt/*β*-catenin signaling pathway performs an important role for the initiation and development of esophagus cancer [11–13]. Once the Wnt/*β*-catenin signaling pathway is overactivated, the patterns of target genes c-MYC and CyclinD1 related to cell proliferation and migration are increased, which promotes cell proliferation and migration, resulting in malignant transformation of cells [14]. In our study, we discovered that the protein levels of *β*-catenin, c-MYC, and CyclinD1 were significantly increased when PEA3 was overexpressed (Figures 5(a)–5(d)). Moreover, siRab8A transfection reduced the protein levels of *β*-catenin, c-MYC, and CyclinD1 and suppressed the effect of PEA3-OE on *β*-catenin, c-MYC, and CyclinD1 expression (Figures 5(a)–5(d)). To further validate the function of the Wnt/*β*-catenin signaling pathway, M435-1279 (Wnt/*β*-catenin inhibitor) was applied. Results from Figures 5(e)–5(h) revealed that siRab8A or M435-1279 treatment reduced the protein levels of *β*-catenin, c-MYC, and CyclinD1, which was more significant when siRab8A and M435-1279 were treated together. Additionally, functional experiments showed that the OD values and clone number of KYSE150 and TE-1 cells were obviously reduced after siRab8A or M435-1279 treatment, especially when siRab8A and M435-1279 were cotreated (Figures 5(i)–5(l)). Based on the above findings, we inferred that Rab8A, transcriptionally regulated by PEA3, promoted the development of esophagus cancer cells by activating the Wnt/*β*-catenin signaling pathway.

## 4. Discussion

The tumor-promoting effect of Rab8A has been involved in various physiological activities and signaling pathways [7]. In this study, we discovered that Rab8A was highly expressed in esophagus cancer samples, and knockdown of Rab8A suppressed the growth, migration, and invasion as well as induced apoptosis. Additionally, PEA3 has been identified as an upstream transcriptional factor of Rab8A and positively regulated Rab8A expression. Moreover, the effect of siRab8A on esophagus cancer cells could be diminished by PEA3 upregulation.

The PEA3 subfamily, as a subgroup of the E26 transformation-specific family, includes ETV1, ETV4, and ETV5. Functionally, the PEA3 subfamily is related to motor coordination, axon guidance, metabolism, neuron development, hormonal regulation, fertility, and tumorigenesis [15]. PEA3, also named ETV4, has been found to be highly expressed in many tumors [15]. High level of PEA3 usually resulted in a more aggressive tumor phenotype and drug resistance [16]. As an oncogenic transcription factor, PEA3 was discovered to directly target to the 5′ and 3′ MYC enhancers, insinuating that PEA3 may modulate the expression of several important oncogenes [17]. The PEA3 transcription factor is usually activated in gastric cancer, hepatocellular carcinoma, colorectal cancer, and lung cancer [18–21]. In esophageal squamous cell carcinoma and esophageal adenocarcinoma, PEA3 overexpression significantly elevated MMP levels and activated metastatic progression [22, 23]. In our study, PEA3 was identified as a transcriptional factor of Rab8A in esophagus cancer. Moreover, PEA3 was highly expressed in esophagus cancer samples, and overexpression of PEA3 promoted the proliferation, migration, and invasion of esophagus cancer cells as well as suppressed apoptosis. Additionally, the function of Rab8A depletion on esophagus cancer cells was reversed by PEA3 upregulation.

The Wnt/*β*-catenin signaling pathway is a conserved signaling axis taking part in various physiological processes including proliferation, apoptosis, differentiation, invasion, migration, and tissue homeostasis [24, 25]. Abnormal Wnt/*β*-catenin signaling pathway promotes tumor stem cell renewal, cell proliferation, and differentiation, thus performing an important role in tumorigenesis and therapeutic response [26]. In the Wnt/*β*-catenin signaling pathway, aberrant regulation of *β*-catenin, which is the crucial component of the Wnt/*β*-catenin signaling pathway, resulted in early events in carcinogenesis [27, 28]. Additionally, the relationship between Rab8A and Wnt pathway has been reported. For example, Rab8A controls Wnt delivery in producing cells and is crucial for Paneth cell maturation [29]; Rab8A attenuates the Wnt signaling pathway and is required for mesenchymal differentiation into adipocytes [30]; Rab8A has been discovered to regulate the development of non-small-cell lung cancer by modulating the Wnt/*β*-catenin signaling pathway [31]. In our study, overexpression of PEA3 increased the protein levels of c-MYC, *β*-catenin, and CyclinD1, while siRab8A transfection diminished the effect of PEA3 overexpression and suppressed the protein levels of c-MYC, *β*-catenin, and CyclinD1. Additionally, the inhibitor of the Wnt/*β*-catenin signaling pathway was applied. We discovered that suppression of the Wnt/*β*-catenin signaling pathway could inhibit the growth ability of esophagus cancer cells.

Several deficiencies in our study should be pointed out. First, our results were achieved only based on cell experiments; animal experiments will be needed to validate the results. Additionally, more molecular mechanism about Rab8A in esophagus cancer should be revealed.

## 5. Conclusions

Taken together, our results showed that knockdown of Rab8A could diminish the growth, invasion, and migration abilities as well as induce the apoptotic ability. Moreover, Rab8A was transcriptionally regulated by PEA3 and interacted with PEA3 to regulate the malignant behavior of esophagus cancer cells. The Wnt/*β*-catenin signaling pathway was positively regulated by Rab8A/PEA3 in esophagus cancer cells. The above results indicated that Rab8A, transcriptionally modulated by PEA3, promoted the growth and metastasis abilities of esophagus cancer cells by activating Wnt/*β*-catenin signaling.

## Figures and Tables

**Figure 1:** Rab8A was highly expressed in esophageal cancer cell lines, and siRab8A transfection significantly reduced Rab8A. (a–c) Results from qPCR and western blotting assays showed that Rab8A was overexpressed in KYSE150, TE-1, and Eca109 cells. (d, e) siRab8A-1 or siRab8A-2 transfection obviously reduced Rab8A expression in KYSE150 and Eca109 cells. ^∗∗^*P* < 0.01 vs. control.

**Figure 2:** siRab8A transfection affected the growth, apoptosis, migration, and invasion abilities of KYSE150 and Eca109 cells. (a, b) The OD values of KYSE150 and Eca109 cells were obviously reduced after siRab8A-1 or siRab8A-2 transfection. (c, d) The number of cell clones in KYSE150 and Eca109 cells was obviously reduced after siRab8A-1 or siRab8A-2 transfection. (e–h) siRab8A-1 or siRab8A-2 transfection obviously reduced Bcl-2 and increased BAK and active caspase-3 in KYSE150 and Eca109 cells. (i–l) The number of cell migration and invasion in KYSE150 and Eca109 cells was obviously reduced after siRab8A-1 or siRab8A-2 transfection. ^∗∗^*P* < 0.01 vs. control.

**Figure 3:** PEA3 was regarded as a transcriptional factor of Rab8A and positively regulated Rab8A expression. (a) In the WT-Rab8A group, overexpression of PEA3 significantly increased the luciferase activity. (b, c) After si-NC or si-PEA3 treatment, ChIP assay was carried out using control IgG or Rab8A antibody. Then, qPCR was performed to analyze Rab8A enrichment. (d–g) In KYSE150 and Eca109 cells, siPEA3 transfection reduced the protein levels of PEA3 and Rab8A; PEA3-OE transfection increased the protein levels of PEA3 and Rab8A. (h, i) Data from western blotting assays showed that Rab8A and PEA3 were highly expressed in esophageal cancer tissues. ^∗∗^*P* < 0.01 vs. normal. T: tumor, N: normal.

**Figure 4:** The biological effects of PEA3-OE on KYSE150 and Eca109 cells were counteracted by si-Rab8A. (a–d) The promoting effects of PEA3-OE on OD values and cell clone numbers in KYSE150 and Eca109 cells were reversed by si-Rab8A treatment. (e–h) PEA3-OE treatment increased Bcl-2 expression and decreased Bak and active caspase-3 expression in KYSE150 and Eca109 cells, whereas the phenomena were reversed by the addition of si-Rab8A. (i–l) The increased invasion and migration abilities of KYSE150 and Eca109 cells caused by PEA3-OE were inhibited by the administration of si-Rab8A. ^∗∗^*P* < 0.01 vs. control; ^#^*P* < 0.05 and ^##^*P* < 0.01 vs. PEA3-OE.

**Figure 5:** The Wnt/*β*-catenin signaling pathway was involved in the regulation of PEA3/Rab8A on KYSE150 and Eca109 cell behaviors. (a–d) Protein levels of c-MYC, *β*-catenin, and CyclinD1 in KYSE150 and Eca109 cells were detected by western blotting after control, PEA3-OE, or PEA3-OE+si-Rab8A treatment, respectively. ^∗∗^*P* < 0.01 vs. control; ^##^*P* < 0.01 vs. PEA3-OE. (e–h) Protein levels of c-MYC, *β*-catenin, and CyclinD1 in KYSE150 and Eca109 cells were detected by western blotting after control, siRab8A, inhibitor, or siRab8A+inhibitor treatment, respectively. (i, j) The OD values in KYSE150 and Eca109 cells were detected by CCK-8 assay after control, siRab8A, inhibitor, or siRab8A+inhibitor treatment, respectively. (k, l) The cell clone number in KYSE150 and Eca109 cells was detected by colony formation assay after control, siRab8A, inhibitor, or siRab8A+inhibitor treatment, respectively. ^∗∗^*P* < 0.01 vs. control; ^##^*P* < 0.01 vs. siRab8A.

## Data Availability

The datasets used and/or analyzed during the current study are available from the corresponding author on reasonable request.
